# Pharmacokinetics of Veratramine and Jervine from Alcohol Extracts of Radix Veratri

**DOI:** 10.1155/2022/8289548

**Published:** 2022-06-23

**Authors:** Song Wang, Jiali Cui, Gaoqiong Zhao, Hongbin Liu, Jingkun Wang

**Affiliations:** ^1^Yunnan Institute of Materia Medica, Kunming, 650111 Yunnan, China; ^2^Yunnan Technology and Business University, 651701, China; ^3^Yunnan Province Company Key Laboratory for TCM and Ethnic Drug of New Drug Creation, 650111, China

## Abstract

**Background:**

*Chinese Materia Medica* and *Jiangsu New Medical College* record that Radix Veratri root is *Liliaceae Veratrum taliense Loses. f.* and the root of *Veratrum stenophyllum Diels*. According to *traditional Chinese medicine* (*TCM*) *example*, Radix Veratri is a Liliaceae plant Veratrum taliense. Another literature pointed out that the aliases of Veratrum taliense and Veratrum angustifolia are both Radix Veratri, and their effects are basically the same. The main active ingredient of Veratrum is veratramine, of which veratramine and Jervine are higher in content, reaching 24.60% and 21.28% of the total alkaloids, respectively. Veratrum alkaloids are both toxic and effective ingredients. In addition to its good clinical efficacy, attention should also be paid to its pharmacokinetic characteristics in vivo. It is particularly important to study the pharmacokinetic characteristics of veratramine and Jervine in vivo.

**Objective:**

The goal of this study was to develop a simple and effective method for measuring veratramine and Jervine in rat plasma at the same time. This method was used to study the pharmacokinetic characteristics of veratramine and Jervine in the alcohol extract of Radix Veratri in rats, to provide a reasonable basis for the clinical use of Radix Veratri.

**Methods:**

Eighteen SD rats were randomly assigned into three groups, half male and half female, and were given 0.04 g/kg, 0.08g/kg, and 0.16 g/kg Radix Veratri alcohol extract, respectively. Blood samples were collected at different time points and were analyzed by LC-MS/MS after protein precipitation. Bullatine was set as the internal standard; the plasma samples were extracted with ethyl acetate. After the sample was processed, acetonitrile-10 mM ammonium acetate, whose pH was adjusted to 8.8 with ammonia water, was taken as the mobile phase. Veratramine quantitative ion pair was 410.1⟶295.1*m*/*z*, Jervine quantitative ion pair was 426.2⟶114.1*m*/*z*, and Bullatine B (IS) quantitative ion pair was 438.2⟶420.1*m*/*z*. In the positive ion mode, the multireaction monitoring (MRM) mode was used to determine the blood concentration of veratramine and Jervine. DAS 3.3.0 was used to calculate the relevant pharmacokinetic parameters.

**Results:**

Veratramine had a good linear relationship in the concentration range of 0.0745~18.2 ng/mL, and that of Jervine was 1.11~108 ng/mL. The correlation coefficient *r* of three consecutive batches of the standard curve was greater than 0.995. Veratramine's lower quantification limit was 0.745 ng/mL, Jervine's was 1.11 ng/mL, and precision and accuracy were both less than 15%. The accuracy of veratramine was between 88.96% and 101.85%, and the accuracy of Jervine was between 92.96% and 104.50%. This method was adopted for the pharmacokinetic study of alcohol extracts of Radix Veratri. The results showed that only *C*_max_ of veratramine female rats did not show linear kinetic characteristics in the dose range of Radix Veratri alcohol extract from 0.04 g/kg to 0.16 g/kg. For AUC_0‐*t*_ and *C*_max_ of veratramine and Jervine, it could not determine whether the Radix Veratri alcohol extract showed linear kinetic characteristics within the dosage range of 0.04 g/kg~0.16 g/kg. Veratramine and Jervine showed obvious gender differences in the absorption and elimination stages. The absorption rate of veratramine and Jervine by male mice was about 10 times higher than that of female mice, and the elimination rate of male mice is about 20 times lower than that of female mice. It was suggested that the clinical application of the steroidal alkaloids veratramine and Jervine in Radix Veratri required rational use of drugs based on gender.

**Conclusion:**

An LC-MS/MS analysis method suitable for the pharmacokinetic study of veratramine and Jervine in Radix Veratri in SD rats was established to provide a basis for in vivo pharmacokinetic studies. The pharmacokinetic characteristics of veratramine and Jervine in the alcohol extract of Radix Veratri were significantly different in female and male rats. During the clinical use of Radix Veratri, it should pay close attention to the obvious gender differences that may occur after the medication.

## 1. Introduction

Radix Veratri is also known as small Veratri, Veratrum, small brown bag, human hair, etc. The taste is bitter, cool in nature, and highly toxic. It has the effects of dispelling blood stasis and swelling, analgesic and hemostasis, lowering blood pressure [1–3], expectorant, and resuscitation. Indications are traumatic injuries, fractures, paraplegia, epilepsy, rheumatic pain, traumatic bleeding, etc., and it is also used to treat cancer in the folk [4–8]. The main active ingredients of Veratrum are steroidal alkaloids, among which the content of veratramine and Jervine is relatively high, reaching 24.60% and 21.28% of total alkaloids, which has antitumor and antibacterial effects [9, 10]. Veratramine and Jervine can specifically bind to the upstream activator of the Hh pathway, Smo, to inhibit the transmission of pathway signals, thereby inhibiting the proliferation effect of tumor cells [11, 12]. Moreover, veratramine and Jervine are also toxic components, and the toxicity is strong, mainly manifested as teratogenicity, reproductive toxicity, etc. [9, 13, 14]. Radix Veratri is used as a special Yi medicine for the treatment of bruises. In addition to its good clinical efficacy, attention should also be paid to its pharmacokinetic characteristics in the body. In particular, the research on the in vivo pharmacokinetic characteristics of compounds that contain both effective and toxic ingredients is particularly important. This work was developed to establish an HPLC-MS/MS method for the determination of veratramine and Jervine in rat plasma, and a systematic methodological verification was conducted. The pharmacokinetic characteristics of veratramine and Jervine in the alcohol extract of Radix Veratri in rats at different dosage levels were systematically studied. The confidence interval method was used for statistical analysis of the obtained pharmacokinetic parameters [15–19]. The dose range in which veratramine and Jervine exhibited linear dynamic characteristics of the dose-exposure level was explored. In addition, the pharmacokinetic parameters of Radix Veratri alcohol extract at different doses were analyzed and compared [5, 20, 21]. The above studies can provide references for the follow-up safety evaluation and clinical medication of veratramine and Jervine.

The paper's organization paragraph is as follows: The materials and methods are presented first. Second are experimental results of the proposed work. Thirdly, it consists of the results and discussion sections. Finally, the research work is concluded.

## 2. Materials and Methods

### 2.1. Chemicals and Reagents

Veratramine and Jervine reference substances' purity was no less than 98%, which were purchased from Nanjing SenBeiJia Biological Technology Co., Ltd. (batch number: SBJ150701, SBJ150625). Bullatine B (internal standard, purity no less than 98%) was purchased from the Beijing Shengshikangpu Chemical Technology Research Institute (batch number: N-019-150906). Heparin sodium (chromatographically pure) was purchased from Aladdin (batch number: C162031). Ammonium acetate (chromatographically pure) was purchased from Aladdin (batch number: k1616041). Methanol (chromatographically pure) was purchased from MERCK (batch number: I0887507 717). Sinopharm Chemical Reagent Co., Ltd. provided analytical pure ethyl acetate (batch number: 20170824). Sichuan Xilong Chemical Co., Ltd. provided the ammonia (analytical pure) (batch number: 150324). The water was ultrapure water made by the Drug Safety Evaluation Center of Yunnan Institute of Materia Medica.

### 2.2. Liquid Mass Spectrometry Instruments and Conditions

The researchers used an API-3200 triple quadrupole tandem mass spectrometer and an electrospray ionisation ion source (ESI). Multiple reaction monitoring (MRM) was used to quantify the sample, which was separated on an Agilent ZORBAX Extend C18 column. The mobile phase was A (10 mmol/L ammonium acetate) and B (acetonitrile), 0-0.2 min, 10% B; 0.2-2 min, 10%-90% B; 2-5 min, 90% B; 5-5.1 min, 90%-10%B; and 5.1-7.5 min, 10%B. The flow rate was 0.4 mL/min, the column temperature was set to 20°C, and the measurement solution was 10 *μ*L. The mass spectrum parameters were as follows: veratramine *m*/*z*: 410.1⟶295.1, Jervine *m*/*z*: 426.2⟶114.1, and Bullatine B *m*/*z*: 438.2⟶420.1. Ion source parameters were as follows: CUR: 20.00 psi, IS: 5,500.00 V, TEM: 500.0°C, GS1: 50.0 psi, GS2: 50.0 psi, CAD: medium, and interface heater(ihe): on.

### 2.3. Preparation of Standard Solutions and Quality Control Samples

5.45 mg and 5.53 mg of veratramine reference substance and 4.96 mg and 5.13 mg Jervine reference substance were taken, two copies each. Methanol was diluted to stock solutions with concentrations of 545 *μ*g/mL, 553 *μ*g/mL, 496 *μ*g/mL, and 513 *μ*g/mL. Diluted with methanol, the concentrations of veratramine were 0.745, 2.24, 6.70, 20.2, 60.5, and 182 ng/mL; those of Jervine standard working fluid were 11.1, 27.8, 69.5, 174, 434, and 1,080 ng/mL; those of veratramine were 0.745, 2.70, 25.6, and 143 ng/mL; and those of Jervine quality control working solution were 1.11, 31.6, 194, and 724 ng/mL. Quality control samples were used for precision, accuracy, matrix effect, recovery, and stability investigations. The same method was used to prepare Bullatine B (IS) internal standard working solution with a concentration of 128 ng/mL, and all working solutions were stored in a refrigerator at 2-8°C.

### 2.4. Preparation of Plasma Samples

10 *μ*L internal standard working solution was added into a 2 mL EP tube, blown and dried with nitrogen at room temperature, and added with 100 *μ*L of plasma sample mixed in vortex for 2 min. Then, 40 *μ*L 25% ammonia water was added and mixed in vortex for 1 min, and 1 mL ethyl acetate was added and mixed in vortex for 3 min and centrifuged at 6,000 r/min at room temperature for 10 min. 600 *μ*L of the supernatant was taken and blown and dried with nitrogen at room temperature. It was reconstituted with 150 *μ*L methanol and mixed in vortex for 2 minutes and centrifuged at 15,000 r/min at room temperature for 10 minutes, and the supernatant was taken for analysis.

### 2.5. Mass Spectrometry Method Validation

#### 2.5.1. Specificity

It was fully verified according to the US Food and Drug Administration's bioanalytical method verification guidelines, as illustrated in Figures 1 and 2. Under the selected chromatographic conditions, the peak times of veratramine, Jervine, and Bullatine B were 3.84 min, 3.81 min, and 3.21 min, respectively. Endogenous substances in plasma did not affect the detection of veratramine, Jervine, and internal standard Bullatine.

#### 2.5.2. Standard Curve and Lower Limit of Quantification

The standard curve was obtained by measuring no less than six points for each compound. The veratramine concentrations were 0.0745, 0.224, 0.670, 2.02, 6.05, and 18.2 ng/mL, respectively. The Jervine concentrations were 1.11, 2.78, 6.95, 17.4, 43.4, and 108 ng/mL, respectively. The lowest detectable concentration was used to define the lower limit of quantification. It was also repeated six times to ensure precision and accuracy. The veratramine standard curve was *y* = 0.291*x* + 17.1 × 10^−4^ (*r* = 0.9965). The Jervine standard curve was *y* = 0.0462*x* − 5.51 × 10^−3^ (*r* = 0.9981). The lower limits of quantification of veratramine and Jervine were 0.0745 and 1.11 ng/mL, respectively, and those of RSD% were 5.49% and 0.12%, respectively.

#### 2.5.3. Precision and Accuracy

The accuracy and precision of intraday (*n* = 6) and intraday (*n* = 6) were determined after four concentrations of quality control samples were measured, those of veratramine were 0.745, 2.70, 25.6, and 143 ng/mL, respectively, and those of Jervine were 1.11, 31.6, 194, and 724 ng/mL, respectively (Table 1). The absolute value of the relative deviation was not higher than 15%, the accuracy of veratramine was 88.96%~101.85%, and that of Jervine was 92.96%~104.50%. The results showed that the accuracy and precision of this method met the requirements of biological sample analysis.

### 2.6. Extraction Recovery Rate and Matrix Effect

The extraction recovery rate of veratramine and Jervine at three concentrations (*n* = 6) was veratramine of 2.70, 25.6, and 143 ng/mL, respectively, and Jervine of 31.6, 194, and 724 ng/mL, respectively. The extraction recoveries of the two compounds were veratramine of 81.22%~94.42% and Jervine of 81.65%~87.98% (Table 2). The matrix had no influence on veratramine, Jervine, or the internal standard Bullatine B, and it had the same effect on each concentration, meeting the pharmacokinetic analysis and detection requirements.

### 2.7. Stability

The stability of plasma samples stored at room temperature and 2-8°C for 48 hours and 5 days at room temperature is illustrated in Table 3. The untreated plasma samples were kept at room temperature for 20 hours and -20°C for 20 hours, 34 days, and 34 days, respectively. Three freeze-thaw cycles were performed to verify the stability (Table 4). Under the above settings, the relative standard deviations were all less than 15%, and the samples were stable enough to meet the requirements of pharmacokinetic analysis and testing.

### 2.8. Pharmacokinetic Studies

#### 2.8.1. Extraction Preparation

Radix Veratri coarse powder was taken, added with six times 65% ethanol and heated under reflux for extraction three times, 1 h each time, and filtered, and then, the filtrates were combined. The ethanol was recovered under reduced pressure, concentrated into a thick paste, dried under reduced pressure at 70°C, and crushed into final products. The contents of veratramine and Jervine in the extract measured by the HPLC-UV method were 2.69% and 1.79%, respectively.

#### 2.8.2. Drug Administration

0.0805 g, 0.1601 g, and 0.3214 g of alcohol extracts were put into a mortar and ground thoroughly. During the grinding, 20 mL of 0.05% sodium carboxymethyl cellulose was added, which was ground to a uniform suspension and placed in a refrigerator at 2~8°C. Each SD rat was given a single dose, and the administration volume was 10 mL/kg. According to this method, the dosage of Radix Veratri alcohol extract was 0.04 g/kg, 0.08 g/kg, and 0.16 g/kg, respectively. The corresponding veratramine doses were 0.108, 0.215, and 0.430 mg/mL, and the Jervine doses were 0.072, 0.143, and 0.286 mg/mL, respectively.

### 2.9. Animal Experiments and Sample Collection

After the ethical approval, a total of 18 healthy SPF SD rats were taken, the license number was SCXK (Sichuan) 2015-030, and the laboratory animal quality certificate number was No. 51203500004128. There are 9 females and 9 males each, 7-8 weeks, the weight range of female rats was 200-230 g, and the weight range of male rats was 200-230 g. The weight difference of the grouped animals was not more than 20% of the average weight of all animals, and they were rolled into low, medium, and high dose groups, with half males and half females. Samples were collected at 0.15, 0.5, 1, 3, 6, 9, 18, 30, 48, 72, and 96 h before intragastric administration (0 h) and after administration. 0.3 mL of blood was collected from the rat's retroorbital venous plexus, placed in a centrifuge tube soaked in 2 mL of heparin sodium, and centrifuged (3,000 rpm/min) for 15 min, and the plasma was frozen and stored at -20°C for testing.

### 2.10. Data Analysis

The pharmacokinetic parameters were calculated using the DAS 3.3.0 pharmacokinetic program to calculate the main pharmacokinetic parameters AUC_0‐*t*_, AUC_0−∞_, and *T*_1/2_. *C*_max_ and *T*_max_ adopted actual measured values, and other pharmacokinetic parameters adopted statistical moment parameters.

Power function model PK = *α* · *D*^*β*^ (*D* was the dose, while *α* and *β* were constants) was used for multidose linear relationship analysis. *α*, *β*, and the 90% confidence interval (90% CI) of the *β* value in the power function model were calculated using the DAS 3.3.0 pharmacokinetic program. The linear judgment interval after the criterion was changed using the DAS 3.3.0 pharmacokinetic program was 0.839-1.161, based on the bioequivalence criterion of 0.8 to 1.25. When the 90% CI of the *β* value fell within the linear judgment interval, the linear relationship was considered to be established; otherwise, the linear relationship did not hold.

## 3. Results

The absorption rate of male mice was higher than that of female mice, and the elimination rate of male mice was lower than that of female mice, showing obvious gender differences in veratramine (Figure 3) and Jervine (Figure 4). At the different doses designed in this experiment, there were obvious gender differences. The drug exposure of veratramine in male rats was much higher than that in female rats. With the increase of the administered dose, the exposure dose of veratramine to both male and female rats also increased. The absorption, distribution, and elimination of veratramine in rats can be affected by some molecules that were inadvertently removed during the extraction process. Furthermore, this effect was more noticeable throughout the stage of drug distribution. Jervine drug exposure was substantially higher in male rats than in female rats. The exposure dose of female and male rats to the Jervine medication increased as the provided dose was increased. Certain compounds that were inevitably extracted during the extraction process can affect the absorption, distribution, and elimination of Jervine in rats. Unlike veratramine, however, this effect was more obvious in the drug elimination phase. The main pharmacokinetic parameters of Radix Veratri alcohol extract low, medium, and high dose groups were analyzed to compare the results (Table 5).

### 3.1. Linear Dynamic Judgment

DAS 3.3.0 was employed, the *Power Model* in the hypothesis test method was used according to the standard of 0.8~1.25, and the linear interval calculated by 1 ± ln(*θL*)/ln(DH/DL) < *β* < 1 ± ln(*θH*)/ln(DH/DL) should be between 0.839 and 1.161. The results of determinations of whether veratramine and Jervine in the alcohol extract of Radix Veratri showed linear kinetic characteristics within the dose range of 0.04 g/kg to 0.16 g/kg are presented in Table 6.

## 4. Discussion

In the initial selection of internal standards, the first selected compounds were aconitine, hypaconitine, Bullatine A, Wilforgine, and Bullatine B. The response of aconitine and hypaconitine could not reach the linear medium concentration, and the response was extremely unstable. Although Bullatine A and Wilforgine could achieve the required response, their chromatographic peaks were far from the target peak, and the analysis time was long, which increased the experimental cost. The peak shape of Bullatine B was good, it can be completely separated from the target peak, and it can be better dissolved in the sample. After testing, there was no Bullatine B in Radix Veratri, so Bullatine B was selected as the internal standard.

*C*_max_ of veratramine female rats did not show linear kinetic characteristics within the dosage range of 0.04 g/kg~0.16 g/kg of Radix Veratri alcohol extract. For others, it cannot be judged whether AUC_0‐*t*_ and *C*_max_ were linear kinetic characteristics within the dosage range of 0.04 g/kg~0.16 g/kg of Radix Veratri alcohol extract.

In the low-dose group, middle-dose group, and high-dose group, the average AUC_0‐*t*_ and average *C*_max_ of males were much higher than those of females. Female rats have considerably greater *CLz*/*F* clearance rates of veratramine and Jervine than male rats. However, there was no discernible variation in the half-life of veratramine in male and female rats, while the half-life of Jervine was considerably different in female and male rats. This was due to the fact that female rats had a considerably higher volume of veratramine dispersion than male rats, and Jervine was removed faster in female rats than in male rats. The above situation showed that after administration of the alcohol extract of Radix Veratri, veratramine and Jervine were more widely distributed in female rats than in male rats, but the clearance rate was much lower than that in female rats. In addition, at the dosage designed in this experiment, the average AUC_0‐*t*_ and average *C*_max_ of males were much higher than that of females. The drug exposure in male rats was much higher than that of female rats, but the clearance rate was much lower than that of female rats. Male rats were more prone to accumulate toxicity in the course of long-term administration, and the symptoms of toxicity were greater than that of females.

## 5. Conclusion

The blood drug concentration and main pharmacokinetic parameters of the Radix Veratri alcohol extract group were analyzed. The absorption rate of veratramine and Jervine by males was higher than that of female rats. Although Bullatine A and Wilforgine were able to provide the desired response, their chromatographic peaks were distant from the intended peak, and the analysis time was considerable, increasing the expense of the experiment. Male mice had a lower elimination rate than female mice, indicating clear gender differences. Finally, the clinical usage of the steroidal alkaloids veratramine and Jervine in Radix Veratri necessitates gender-based medication selection.

## Figures and Tables

**Figure 1:** (a) Total ion current diagram of blank plasma plus veratramine *m*/*z*: 426.2/114.1, Jervine *m*/*z*: 426.2/114.1, and Bullatine B *m*/*z*: 438.2/420.1; (b) the ion current diagram of extracted veratramine *m*/*z*: 410.1/295.1; (c) the ion current diagram of extracted Jervine *m*/*z*: 426.2/114.1; (d) the ion current diagram of extracted Bullatine B *m*/*z*: 438.2/420.1.

**Figure 2:** (a) Total ion current diagram of 1 h unknown concentration of plasma sample of formal experiment No. 22 rat; (b) the ion current diagram of extracted veratramine *m*/*z*: 410.1/295.1; (c) the ion current diagram of extracted Jervine *m*/*z*: 426.2/114.1; (d) the ion current diagram of extracted Bullatine B *m*/*z*: 438.2/420.1.

**Figure 3:** (a) Female and male average drug-time curve of 0.04 g/kg VER; (b) female and male average drug-time curve of 0.08 g/kg VER; (c) female and male average drug-time curve of 0.16 g/kg VER; (d) VER female average drug-time curve; (e) VER male average drug-time curve.

**Figure 4:** (a) Female and male average drug-time curve of 0.04 g/kg JER; (b) female and male average drug-time curve of 0.08 g/kg JER; (c) female and male average drug-time curve of 0.16 g/kg JER; (d) JER female average drug-time curve; (e) JER male average drug-time curve.

**Table 1:** Precision and accuracy.

Compound	Concentration (ng/mL)	Accuracy (RE%)	Intraday precision (RSD%)	Daytime precision (RSD%)
VER	0.745	96.51	06.54	09.21
	02.70	98.52	06.02	97.78
	25.6	95.70	05.31	99.22
	143	96.71	11.93	94.62

JER	01.11	102.70	07.11	100.18
	31.6	100.32	08.52	99.05
	194	101.10	04.08	102.20
	724	92.96	13.19	94.61

**Table 2:** Extraction recovery rate and matrix effect.

Compound	Concentration (ng/mL)	Recovery rate (%) (±SD)	Matrix effect (%) (±SD)
VER	2.70	94.42 ± 0.01	116.22 ± 13.10
	25.60	81.22 ± 0.06	117.08 ± 8.26
	143	93.29 ± 0.26	110.44 ± 8.02

JER	31.60	87.98 ± 0.01	137.15 ± 15.86
	194	81.65 ± 0.07	143.50 ± 5.02
	724	84.90 ± 0.22	130.63 ± 7.46

**Table 3:** Stability of plasma samples after treatment.

Compound	Conditions					
	Room temperature 48 h		2~8°C 48 h		Room temperature 5 d	
	Accuracy	RSD%	Accuracy	RSD%	Accuracy	RSD%
VER	-2.22%	6.44%	6.30%	5.92%	5.19%	4.93%
	-4.69%	5.47%	-0.39%	5.10%	3.12%	7.20%
	-4.90%	13.01%	-1.40%	7.16%	0.70%	9.44%

JER	0.95%	9.31%	7.91%	8.27%	-1.27%	8.91%
	-5.46%	4.53%	4.12%	7.26%	-9.79%	3.20%
	-0.81%	14.70%	-3.18%	9.67%	-11.60%	2.09%

**Table 4:** Stability of plasma samples before treatment.

Compound	Conditions							
	Room temperature 20 h		-20°C 20 h		-20°C 34 d		-20°C 34 d freeze-thaw three times	
	Accuracy	RSD%	Accuracy	RSD%	Accuracy	RSD%	Accuracy	RSD%
VER	7.41%	8.62%	8.15%	12.67%	2.59%	10.47%	-5.92%	7.48%
	3.52%	5.66%	3.52%	10.19%	-3.52%	10.12%	-1.17%	6.72%
	2.80%	10.48%	10.49%	12.53%	10.49%	11.93%	-1.40%	5.53%

JER	7.91%	4.16%	14.87%	10.22%	-4.11%	10.59%	0.63%	8.43%
	-0.21%	4.80%	-0.52%	11.66%	-2.06%	5.78%	-3.61%	7.70%
	-1.10%	14.28%	2.35%	11.40%	-7.46%	4.10%	-5.39%	5.08%

**Table 5:** Comparison of main pharmacokinetic parameters of Radix Veratri alcohol extract.

Compound	Group	Gender	*C*_max_	*T*_max_	*T*_1/2_	AUC_0‐*t*_ (*μ*g/L∗h)	AUC_0-∞_ (*μ*g/L∗h)	MRT_0‐*t*_ (h)	MRT_0-∞_ (h)	*Vz*/*F* (L/kg)	*CLz*/*F* (L/h/kg)
VER	—	♀♂	10.8 ± 10.3	1.83 ± 1.29	3.71 ± 0.917	81 ± 83	82 ± 83	4.88 ± 1.88	5.63 ± 0.583	14779 ± 15974	3234 ± 3421
			18.7 ± 21.8	5.25 ± 3.74	7.25 ± 3.08	220 ± 543	225 ± 246	8.70 ± 2.49	10.63 ± 3	29509 ± 34086	3948 ± 5244
			24.5 ± 26.8	7.42 ± 11.51	14.26 ± 11.94	488 ± 594	492 ± 591	15.68 ± 5.4	22.19 ± 15.25	54120 ± 72536	2365 ± 2541
	0.04 g/kg	♀	1.40 ± 0.735	2.17 ± 1.44	3.06 ± 0.80	6 ± 2	7 ± 2	3.84 ± 0.19	5.26 ± 0.55	27931 ± 10901	6211 ± 637
	0.08 g/kg		1.38 ± 0.208	5.17 ± 4.31	6.04 ± 4.08	11 ± 5	13 ± 6	6.75 ± 0.81	9.77 ± 4.16	56524 ± 26712	7699 ± 5153
	0.16 g/kg		1.93 ± 0.717	3.50 ± 4.77	18.23 ± 16.93	30 ± 9	38 ± 12	15.32 ± 3.98	28.24 ± 20.38	105156 ± 73053	4509 ± 1528
	0.04 g/kg	♂	20.2 ± 0.939	1.50 ± 1.32	4.35 ± 0.46	157 ± 17	157 ± 17	5.92 ± 0.44	6.01 ± 0.35	1628 ± 367	257 ± 30
	0.08 g/kg		36.1 ± 16.8	5.33 ± 4.04	8.46 ± 1.62	429 ± 127	436 ± 130	10.65 ± 1.85	11.49 ± 1.73	2495 ± 1303	197 ± 71
	0.16 g/kg		47.1 ± 16.5	11.33 ± 16.20	10.28 ± 4.72	946 ± 502	947 ± 503	16.05 ± 7.52	16.14 ± 7.50	3084 ± 1742	221 ± 152

JER	—	♀♂	26.6 ± 26.2	0.71 ± 0.33	11.10 ± 16.86	196 ± 193	218 ± 179	5.28 ± 1.24	16.30 ± 24.25	6571 ± 8482	606 ± 711
			45.2 ± 51.2	4.33 ± 4.17	20.08 ± 24.28	572 ± 550	660 ± 500	11.96 ± 4.65	30.35 ± 34.43	6270 ± 6922	240 ± 232
			44.9 ± 45.1	8.25 ± 11.13	29.47 ± 41.47	1100 ± 1225	1361 ± 1462	14.03 ± 5.07	45.08 ± 58.76	16572 ± 19840	501 ± 579
	0.04 g/kg	♀	3.64 ± 1.59	0.58 ± 0.38	17.49 ± 24.18	20 ± 5	57 ± 51	4.18 ± 0.38	25.77 ± 34.65	12439 ± 8746	1106 ± 717
	0.08 g/kg		7.72 ± 2.79	3.33 ± 4.91	30.91 ± 33.43	113 ± 78	258 ± 156	11.61 ± 7.15	46.79 ± 46.33	11453 ± 6244	401 ± 239
	0.16 g/kg		6.16 ± 4.15	5.17 ± 4.31	46.30 ± 58.01	86 ± 36	264 ± 230	10.94 ± 1.62	68.22 ± 83.70	31977 ± 16494	922 ± 553
	0.04 g/kg	♂	49.5 ± 11.9	0.83 ± 0.29	4.61 ± 1.22	372 ± 17	378 ± 17	6.38 ± 0.25	6.83 ± 0.75	703 ± 108	106 ± 5
	0.08 g/kg		82.8 ± 48.3	5.33 ± 4.04	9.26 ± 2.17	1032 ± 344	1063 ± 337	12.32 ± 1.61	13.92 ± 2.54	1087 ± 458	80 ± 21
	0.16 g/kg		83.6 ± 23.6	11.33 ± 16.20	12.64 ± 9.24	2114 ± 816	2459 ± 1296	17.13 ± 5.73	23.37 ± 10.91	1168 ± 381	80 ± 46

**Table 6:** Judgment and statistics of the linear kinetic relationship between veratramine and Jervine in the alcohol extract of Radix Veratri.

Compound	Gender	Pharmacokinetic parameters	*α*	*β*	*r* (correlation coefficient)	Judgment interval	Beta value 95% confidence interval	Judgment result
VER	Female	AUC_0‐*t*_	5.465	1.186	0.88	0.839-1.161	0.613-1.759	Fail to judge
		*C*_max_	1.083	0.274	0.428	0.839-1.161	-0.243-0.792	No
	Male	AUC_0‐*t*_	8.996	1.212	0.889	0.839-1.161	0.654-1.770	Fail to judge
		*C*_max_	4.912	0.581	0.768	0.839-1.161	0.148-1.014	Fail to judge

JER	Female	AUC_0‐*t*_	6.558	1.026	0.692	0.839-1.161	0.069-1.984	Fail to judge
		*C*_max_	2.472	0.333	0.357	0.839-1.161	-0.446-1.112	Fail to judge
	Male	AUC_0‐*t*_	9.863	1.210	0.933	0.839-1.161	0.793-1.627	Fail to judge
		*C*_max_	5.14	0.374	0.544	0.839-1.161	-0.141-0.888	Fail to judge

## Data Availability

The datasets used during the current study are available from the corresponding author on reasonable request.
